The article "Anti-Diabesity Middle Eastern Medicinal Plants and Their Action Mechanisms" was published in 2022. Journal: Evid Based Complement Alternat Med.

# Anti-Diabesity Middle Eastern Medicinal Plants and Their Action Mechanisms

**DOI:** 10.1155/2022/2276094

**Published:** 2022-07-18

**Authors:** Bashar Saad, Abdalsalam Kmail, Sameena Z. H. Haq

**Affiliations:** ^1^Faculties of Medicine and Arts and Sciences, Arab American University, P.O. Box 240, Jenin, State of Palestine; ^2^Al-Qasemi Research Center, Al-Qasemi Academy, P.O. Box 124, Baqa El-Gharbia 30100, Israel; ^3^Foundation for Science Technology and Civilisation, Manchester, UK

## Abstract

Over the last four decades, the escalation in diabetes and obesity rates has become epidemic all over the world. Diabesity describes the strong link between T2D and obesity. It correlates deeper with the elevated risks of developing cardiovascular disease hypertension, stroke, and several malignancies. Therapeutic usage of medicinal plants and natural products in the treatment of diabetes and obesity has long been known to physicians of Greco-Arab and Islamic medicine. Improved versions of their abundant medicinal plant-based formulations are at present some of the most popular herbal treatments used. Preclinical and clinical data about medicinal plants along with their bioactive constituents are now available, justifying the traditionally known therapeutic uses of products derived from them for the prevention and cure of obesity-related T2D and other health problems. The aim of this review is to systematize published scientific data dealing with the efficiency of active ingredients or extracts from Middle Eastern medicinal plants and diet in the management of diabesity and its complications. Google Scholar, MEDLINE, and PubMed were searched for publications describing the medicinal plants and diet used in the management of T2D, obesity, and their complications. The used keywords were “medicinal plants” or “herbals” in combination with “obesity,” “diabetes,” “diabetes,” or nephropathy. More than 130 medicinal plants were identified to target diabesity and its complications. The antidiabetic and anti-obesity effects and action mechanisms of these plants are discussed here. These include the regulation of appetite, thermogenesis, lipid absorption, and lipolysis; pancreatic lipase activity and adipogenesis; glucose absorption in the intestine, insulin secretion, glucose transporters, gluconeogenesis, and epigenetic mechanisms.

## 1. Introduction

Diabesity is a term used to describe the combined adverse health effects of obesity and type 2 diabetes (T2D) [1, 2]. A large number of clinical trials confirm the link between being overweight and the higher risk for the development of T2D [3–7]. The rate of T2D increases with the degree of excess weight 3-fold and 20-fold with a body mass index (BMI) of 25.0–29.9 kg/m^2^ and over 30 kg/m^2^, respectively [4]. In particular, abdominal fat accumulation deteriorates insulin resistance, hence a strong, independent risk of developing T2D [8] (Figure 1). Obesity has reached epidemic levels throughout the globe, and it is now considered as one of the main lifestyle diseases. According to the World Health Organization (WHO), worldwide obesity has nearly tripled since 1975. In 2016, 39% (1.9 billion) of adults aged 18 years and over were overweight, and 13% (650 million) were obese. More than 340 million children and 5–19-year-old teenagers were overweight or obese. In 2020, 39 million children (under 5 years) were overweight or obese [9–12].

The article "Anti-Diabesity Middle Eastern Medicinal Plants and Their Action Mechanisms" was published in 2022. Journal: Evid Based Complement Alternat Med.

In 2013, it was reported that in developing countries such as Malaysia, about 44% and 12% of the adult males were overweight and obese, respectively. Similar prevalence occurs in the East Mediterranean and North African countries. In the Arabian Peninsula, changes in food intake, socioeconomic and demographic factors, decreased physical activity, and a high number of pregnancies all contribute to the rise in overweight and obesity, where the prevalence of obesity in children and teenagers ranges from 3% to 18% in females and 5% to 14% in males [9–12]. Similarly, the incidence of T2D has reached epidemic proportions in these countries.

Globally, the expected number of T2D patients in 2000 was to reach 366 million by the year 2030 [13]; however, according to the International Diabetes Federation (IDF), these estimates were reached early in 2011 [14]. Saudi Arabia, the United Arab Emirates, Bahrain, Kuwait, and Oman were among the 10 countries of the world with the highest reported rates of T2D, namely, 17.7%, 17.3%, 16.5%, 15.7%, and 12.6%, respectively. Over the past three decades, due to the discovery of oil and natural gas, these countries have experienced rapid economic growth and infrastructure development. As a result, T2D has become a serious public health burden because it imposes a substantial strain on individuals as well as on the health systems in these countries [15].

Since T2D and obesity play a significant role in the development of cardiovascular disease (CVD), hypertension, and cancer, their effects from a public health point of view are immense and are in continuous elevation. Thus, we will focus our research efforts on elucidating the aetiology of obesity and diabetes, as well as the processes that trigger the onset of T2D-related comorbidity. Furthermore, we will focus both our public health and clinical efforts on illness prevention and treatment [16–24].

The attempts to identify new genetic obesity susceptibility variants have limited success so far, and the common obesity susceptibility variants identified only clarify a small part of the individuals' variation in risk. Recently, epigenetic factors have been suggested to have a major impact on the existing epidemic of obesity and diabetes. Recent reports suggest that metabolic regulation during adulthood, besides compelling a good equilibrium between energy intake and energy expenditure, is affected by pre- and postnatal environments. Indeed, maternal nutritional constriction during pregnancy can modify the metabolic phenotype of the offspring by means of epigenetic regulation of specific genes, which can be passed to the next generations. Investigations concentrated on epigenetic indices in obesity showed changed methylation and/or histone acetylation levels in genes involved not only in specific but also in more general metabolic pathways [25, 26].

The article "Anti-Diabesity Middle Eastern Medicinal Plants and Their Action Mechanisms" was published in 2022. Journal: Evid Based Complement Alternat Med.

Augmented levels of visceral adiposity and lipid infiltration in the liver and muscle are linked with the development of insulin resistance and T2D. This occurs when the capacity of adipocytes to store fat is overrun [27, 28]. Raised free fatty acid (FFA) concentrations and their conversion to long chain acetyl CoA derivatives lead to decreased insulin signaling, glucose transport, and insulin resistance in the muscle [29]. These FFA-induced alternations lead to “lipotoxicity.” Lipotoxicity in turn induces oxidative stress which may be a factor in the reduction of vital *β*-cell associated with the serum leptin and cytokine concentrations which contribute to *β*-cell damage [30]. Reduced plasma levels of adiponectin, an adipocytokine associated with insulin sensitization and vascular protection, are characteristic of diabesity patients [31]. Elevated levels of circulating resistin (or “resistance to insulin,” originally described as an adipocyte-specific hormone) are a crucial link between obesity and insulin resistance (T2D) [32]. In summary, the contributions of elevated adiposity to elevated levels of FFA, lipid accumulation, and pathogenic patterns of adipokines secretion, particularly in the context of clinical trials, indicate that moderate weight reduction inhibits conversion to T2D in many at-risk persons [33].

T2D is a progressive multifactorial metabolic disease, which is the result of metabolic imbalances, in particular abnormal insulin production, elevated insulin resistance, high glucagon secretion, and drop in viable *β*-cell content [34]. Insulin secretion, as a response to elevated blood glucose levels, is decreased by about 27% in persons with impaired glucose tolerance (IGT) and continues to deteriorate as T2D advances. Untreated hyperglycemia leads to pancreatic *β*-cell destruction, glucose intolerance, and prediabetes. By the time the diagnosis of T2D occurs, half of a patient's *β*-cell viability will have typically lost [35]. T2D is one of the main causes for elevated risk of developing a broad range of pathogenic conditions, including macrovascular disorders (e.g., CVD, stroke), microvascular disease (e.g., retinopathy, neuropathy, nephropathy), and hypertension [19]. Up to three-quarters of T2D patients also have hypertension, and patients with hypertension alone often indicate insulin resistance. Thus, hypertension and diabetes are interconnected complications that share a significant overlap in underlying risk factors, not forgetting any other complications. Similarly, obesity increases the risk of a many chronic diseases, such as coronary heart disease, hyperlipidemia, hypertension, stroke, and certain cancers [1, 19]. It is also linked to the development of additional comorbidity that can further complicate disease treatment, including mobility problems associated with osteoarthritis, obstructive sleep apnea syndrome, and clinical depression. These complications include microvascular and macrovascular disorders. Given the strong association between being overweight and T2D, weight loss in people with prediabetes or diabetes should be a prime aim in therapy plans [1].

The article "Anti-Diabesity Middle Eastern Medicinal Plants and Their Action Mechanisms" was published in 2022. Journal: Evid Based Complement Alternat Med.

Notwithstanding the impressive advancement in synthetic drugs, plant-derived active compounds still make an essential spring of new medicines. They have long been a fruitful source for the discovery of novel medications, finding utility among the popular alternative medicines due to their chemical variety and ability to interact with various biological targets [36]. Presence of various secondary metabolites in plant-based medicines results in a synergistic effect by their action on different cellular targets, thus offering advantages over synthetic drugs, which use only a single compound. Around 80% of the world's population still uses herbal-based extracts and medications as their primary source of therapy. Approximately 25% of presently used pharmaceuticals are herbal in origin or involve at least one active component originating from herbs or chemically modified phytochemicals [36]. In addition, about three-quarters of plants that provide active compounds for pharmaceuticals were discovered because of their use in traditional medicine [26, 37–39].

## 2. Anti-Obesity Therapeutic Potential of Medicinal Plants and Their Active Compounds

### 2.1. Medicinal Plants

Obesity represents a serious disease worldwide. Excessive weight gain results in the development of several chronic diseases such as T2D, nephropathy, hypertension, and cardiovascular diseases. Current pharmacological strategies for the treatment of obesity include reducing diet absorption, reducing fat metabolism, controlling adipose signals, and modulating the satiety center. To slow the progression of overweight/obesity, most strategies focus on dietary and lifestyle improvements, such as limiting calorie consumption and increasing physical activity. However, if these strategies are unsuccessful, anti-obesity drugs are prescribed. As synthetic pharmaceuticals are moderately successful in treating obesity and its associated complications, there is a continuous need to search for newer alternatives to anti-obesity drugs with long-term efficacy and fewer side effects. Medicinal plants produce an enormous number of secondary metabolites that have been found to have beneficial anti-obesity effects (Figure 2). Traditional medical systems-based anti-obesity modalities are diet-based therapies or herbal-based medications. Crude extracts of single plant and plant mixtures, as well as isolated phytochemicals, are some of them. Anti-obesity and antioxidant effects are induced on the metabolism and fat oxidation within the body by herbal-based therapies comprising a wide variety of ingredients. Medicinal plants have been investigated and reported to be beneficial in the management of obesity, diabetes, and other chronic diseases [12, 40–43].

The article "Anti-Diabesity Middle Eastern Medicinal Plants and Their Action Mechanisms" was published in 2022. Journal: Evid Based Complement Alternat Med.

The common opinion that herbal medicines are safe and efficient is not always the case for particular types of people or when consuming random amounts of herbal medicines prescribed. In fact, it is due to such remedies becoming principally appealing to users that they forget to honor dosage, time, etc., which can potentially cause more harm. Despite the lack of control on some of the products, few cases highlight possible side effects [42–47]. Despite the fact that the Food and Drug Administration (FDA) banned *Ephedra sinica* in 2004, it is still available for purchase on the Internet. Moreover, adulteration remains the main problem; hence, quality control should be emphasized [42–47].

A large number of studies have confirmed the anti-obesity effects of several edible herbs, fruits, vegetables, spices, legumes, edible flowers, and mushrooms [26, 36]. Hence, they are potential candidates for the prevention and management of obesity. Controlling appetite and thermogenesis, inhibiting pancreatic lipase activity or adipogenesis, (Figure 1) encouraging lipolysis, modifying gut microbiota, and improving obesity-related inflammation are major anti-obesity targets of phytochemicals [1, 12, 26, 36, 43–48]. A trend in the development of novel anti-obesity medications is to target the adipocyte life cycle with various nutritional bioactivities that influence different phases of the adipocyte life cycle. In this regard, various herbal-derived active ingredients, such as ajoene, apigenin, capsaicin, genistein, kaempferol, luteolin, myricetin, omega-3 fatty acid, quercetin, and resveratrol, influence adipocytes at different phases of development, producing either adipogenesis suppression or apoptosis induction [25, 26]. Moreover, epigenetic pathways (acetylation, methylation, miRNAs, ubiquitylation, phosphorylation, and chromatin packing) are being investigated as possible targets for the development of herbal anti-obesity medicines (Figures 3 and 4).

The article "Anti-Diabesity Middle Eastern Medicinal Plants and Their Action Mechanisms" was published in 2022. Journal: Evid Based Complement Alternat Med.

The group of Ali-Shtayeh [49] evaluated the antioxidant and the pancreatic lipase inhibiting enzyme activities of 90 Palestinian medicinal plants. They reported that approximately 50% of the plant extracts inhibited lipase activity. In fact the most active antioxidant extracts were from *Camellia sinensis, Ceratonia siliqua, Curcuma longa, Sarcopoterium spinosum*, and *Mentha spicata* with IC50 values of 0.5, 0.8, 0.8, 1.2, and 1.2 mg/mL, respectively.

Table 1 summarizes the main anti-obesity medicinal plants and their biochemical action mechanisms. Google Scholar, MEDLINE, and PubMed were used to identify publications describing the medicinal plants and diet used for the treatment of diabetes, obesity, and their complications.

### 2.2. Anti-Obesity Phytochemicals

Recent studies reveal that herbs and their phytochemicals have the power to help people lose weight, either individually or in combination. Multiple phytochemical combinations have synergistic action, which amplifies their therapeutic effects at the molecular, cellular, metabolic, and temporal levels, giving them an edge over chemically manufactured medications Figure 2. Terpenoids, phenolics, and alkaloids are the three primary types of plant active compounds, each with exponentially increasing therapeutic and preventive properties [12, 25, 26, 44].

Terpenoids are one of the most diverse groups of secondary metabolites, with over 20,000 phytochemicals classified under the category “isoprenoids.” Many terpenoids have been reported for their potential as pharmaceuticals. Artemisinin, an antimalarial agent, and taxol, an anticancer drug, are really just examples of terpenoids (Figure 2). The activity of ligand-dependent transcription factors is modulated by the mechanism of action of many terpenoids. Peroxisome proliferator-activated receptors (PPARs) are an example of dietary lipid sensors that manage energy balance. It has been reported that consuming these terpenoids on a daily basis might improve the management of a variety of obesity-related metabolic disorders. Hyperlipidemia, type 2 diabetes, and cardiovascular ailments are examples of diseases that respond well to such intervention [12, 25, 26, 44].

The article "Anti-Diabesity Middle Eastern Medicinal Plants and Their Action Mechanisms" was published in 2022. Journal: Evid Based Complement Alternat Med.

Polyphenols are the second largest category of secondary metabolites, including over 8,000 different polyphenolic molecules identified so far. Flavonoids and non-flavonoids, like tannins, are the two categories of polyphenols [44]. Adipocyte viability and preadipocyte proliferation have been demonstrated to be dramatically inhibited by polyphenolic active substances at the cellular and molecular levels. Polyphenolics also have an anti-inflammatory influence by inhibiting adipocyte differentiation, lipid buildup, and inflammation. Lipolysis and fatty acid oxidation are both stimulated by polyphenols.

Polyphenols have been shown in animal studies to play a vital role in lowering obesity and animal weight, as well as triglycerides, by promoting fat usage and energy expenditure, as well as regulating glucose homeostasis. Importantly, human research yielded mixed outcomes in terms of anti-obesity efficacy. Variations in experimental participants, trial design, length, and chemical forms might be the cause of variations in the results. More work on these parameters (particularly utilizing randomized controlled trials) might lead to more definitive conclusions on the therapeutic value of herbal-derived polyphenols [1, 25, 26, 44].

Lately, different investigations have established that dietary polyphenols can play an essential role in the management of obesity and obesity-related chronic disorders (Figure 2). Green tea catechins, including epigallocatechin gallate (EGCG), curcumin, and resveratrol, which are regularly and historically utilized dietary ingredients across the world, are effective in reducing obesity and obesity-related inflammation. Obesity is controlled using phenolics in both a preventive and a therapeutic manner. They are among the most promising polyphenols, with a wide range of molecular structures and multifactorial consequences. Dietary intervention with these phenolics appears to be promising [12, 25, 26, 44, 50].

Polyphenolic compounds, on the other hand, are found in a wide range of foods, including fruits, vegetables, grains, legumes, and medicinal plants. Polyphenolic compounds, including grape seed proanthocyanidin extract, xanthohumol, genistein, daidzein, cyanidin, apigenin, luteolin, kaempferol, myricetin, quercetin, and epigallocatechin gallate, have been shown to have anti-obesity properties in in vitro, animal, and clinical trials (EGCG). Similarly, coumarin derivatives like esculetin and fucoxanthin, as well as phytoalexins like resveratrol, have been used in carotenoid research to examine their impact on lipid metabolism. Phytosterols, polyunsaturated fatty acids, and organosulfur compounds are further bioactive dietary components with anti-obesity potential [26, 44].

The article "Anti-Diabesity Middle Eastern Medicinal Plants and Their Action Mechanisms" was published in 2022. Journal: Evid Based Complement Alternat Med.

Polyphenols have also been proposed as antioxidants and scavengers of peroxyl and superoxide radicals. They have a role in the control of excessive reactive oxygen species (ROS) and, as a result, in obesity-related diseases by alleviating obesity-related oxidative stress [1, 50]. Polyphenols' antioxidant properties have also been shown to protect against chronic inflammation [50]. Polyphenols have been shown to regulate transcription factors involved in lipid and glucose homeostatic metabolism (e.g., AMPK, PPARs, and SREBP-1c) [50]. Polyphenols' modes of action have been known for having pleiotropic consequences which might involve signal transduction pathways including CCAAT/enhancer binding protein *α*, peroxisome proliferator-activated receptor *γ*, adenosine-monophosphate-activated protein kinase, peroxisome proliferator-activated receptor gamma coactivator 1-alpha, sirtuin 1, sterol regulatory element binding protein-1c, uncoupling proteins-1 and -2, and NF-*κ*B which have a role in adipogenesis, antioxidant defense, and anti-inflammatory responses [1, 26, 50].

Alkaloids are a broad range of secondary metabolites found in herbs. Almost all plants, as well as mammals, fungi, and bacteria, synthesize them (although in minute quantities). Even though most alkaloids are toxic to other animals, they have a wide range of therapeutic effects (Figure 2). They are structurally varied and, unlike other phytochemicals, cannot be grouped into a single chemical group. They also have a profound effect on metabolism. Alkaloids have pharmacological effects on practically every bodily system: coffee stimulates the nervous system; ricinine has cytotoxic effects on the digestive system, causing severe irritation as well as diarrhea and vomiting (typical manifestations). Blood vessels are also targeted by alkaloids [1, 25, 26, 44].

Herbs and their derivatives were shown to have the ability to control appetite, inhibit pancreatic lipase activity, stimulate thermogenesis and lipid metabolism, increase satiety, promote lipolysis, regulate adipogenesis, and induce apoptosis in adipocytes [26, 36]. Additionally, addressing the adipocyte life cycle with diverse dietary bioactives that influence distinct phases of the adipocyte life cycle is an important focus in the development of novel anti-obesity drugs. In this regard, preadipocytes, developing preadipocytes, and mature adipocytes are among the steps of adipocyte development that are targeted by anti-obesity drugs. Capsaicin, genistein, apigenin, luteolin, kaempferol, myricetin, quercetin, docosahexaenoic acid, quercetin, resveratrol, and ajoene are examples of herbal-derived active compounds that affect adipocytes during specific stages of development, resulting in either adipogenesis inhibition or apoptosis induction. Despite the fact that various molecular targets for both therapy and prevention of obesity have been established, single-cell receptor or pathway targeting has had poor success. Furthermore, phytochemical epigenetic mechanisms (acetylation, methylation, miRNAs, ubiquitylation, phosphorylation, and chromatin packing), as well as their preventive and therapeutic implications, have been documented [26, 44].

The article "Anti-Diabesity Middle Eastern Medicinal Plants and Their Action Mechanisms" was published in 2022. Journal: Evid Based Complement Alternat Med.

## 3. Antidiabetic Therapeutic Potential of Medicinal Plants

Despite the great progress made in the treatment of diabetes with insulin and conventional antidiabetic drugs, their therapeutic results are still far from perfect. Drug resistance, adverse effects, and even toxicity are the main side effects of these drugs. For instance, the efficacy of sulfonylureas is lost after 6 years of treatment in 44% of T2D patients, whereas hypoglycemic drugs are ineffective in treating hyperlipidemia [49]. Hence, herbal-derived active compounds represent a potential for detecting promising chief candidates and playing an imperative role in the upcoming drug elaboration programs [1, 26, 31, 34–36, 44, 50–53]. The percentage of T2D patients who use alternative therapies is estimated to be 30.1% in Saudi Arabia, 21% in Lebanon, 41% in Turkey, 41.7% in Egypt, and 39.3% in the United Arab Emirates [15]. However, studies around the world that examined the use of alternative therapies by T2D patients have notably different results ranging from 17 to 72.8% [54].

As previously mentioned, herbs produce a vast number of secondary metabolites which are responsible for health beneficial activities of medicinal plants. Phytochemicals like flavonoids, terpenoids, saponins, carotenoids, alkaloids, and glycosides were found to possess antidiabetic activities [25, 44]. The synergistic action of herbal active compounds (i.e., polyphenols, carotenoids, lignans, coumarins, glucosinolates, etc.) leads to the health beneficial properties of each plant matrix, and this can represent the first step for understanding their medical actions and beneficial activities. Generally, the main approaches to study [25] the synergistic action of phytochemicals are as follows: (1) model system development of interactions [53]; (2) study of extractable and non-extractable compounds [25, 53]; or (3) characterization of biologically active compound-rich extracts [53].

The article "Anti-Diabesity Middle Eastern Medicinal Plants and Their Action Mechanisms" was published in 2022. Journal: Evid Based Complement Alternat Med.

Antidiabetic phytochemicals are classified according to their hypoglycemic action mechanisms; these include principal enzymes in glucose metabolism, cell-surface receptors (e.g., IRS, TM7), glucose transporters (e.g., GLUT2, GLUT4), and signal transduction [25, 53, 55, 56]. The latter represents a potential target for herbal antidiabetic drugs. The antidiabetic activity of whole plant and its crud extracts are mediated through several mechanisms: increased pancreatic insulin secretion via pancreatic augmentation, inhibition of glucose production in the liver and increased glucose uptake in muscle and adipose tissues, inhibition of intestinal glucose absorption, and prevention of diabetes-related complications [26]. Since much of the focus has been on the aerial plant parts, there have been only a few review studies that have focused on the natural compounds found in plant roots that have health advantages. A recent review article [57] has focused on antidiabetic effects of root and rhizome extracts on diabetic mice or rats provoked by streptozotocin or alloxan. According to that literature review, the majority of phytochemicals with antidiabetic bioactivity in the plant root system are engaged in the treatment of diabetes by lowering hyperglycemia and hyperlipidemia, inhibiting glucosidase, and regulating insulin secretion. However, because there are few *in vivo* studies of purified phytochemicals from root extracts, plant root active compounds constitute a largely unstudied promising source of new natural compounds with antidiabetic activities. Flavonoids, phenolic compounds, alkaloids, and phytosteroids are the most common chemical elements in the root system with antidiabetic activities, according to a literature review [57]. Moreover, the root extracts of the plant families Fabaceae, Araliaceae, Asparagaceae, Asteraceae, and Zingiberaceae are regarded as having the most natural antidiabetic constituents [57].

Herbal-based drugs can target signaling cascades involved in glucose homeostasis (e.g., insulin-dependent protein kinase B and insulin-independent AMP-activated protein kinase) or modulate (e.g., allosteric, reversible noncovalent modulation) regulators involved in glucose metabolism [25, 53, 55, 56]. These include reducing intestinal glucose absorption, enhancing insulin secretion, stimulating glucose uptake by tissues, decreasing gluconeogenesis, increasing pancreatic tissue regeneration, and epigenetic mechanisms [26].

DNA methyltransferases and histone-modifying enzymes (e.g., histone deacetylases, histone acetyltransferases, protein arginine methyltransferases, histone methyltransferases, and histone demethylases) are the main epigenetic factors linked to diabetes. In recent years, epigenetic drugs that target the aforementioned enzymes have gained increased interest in treating diabetes and obesity [26]. Many epigenetic drugs are now already in the phase of clinical trials for the management of T2D [26]. Recently, medicinal plants (Table 1) and phytochemicals, such as resveratrol, curcumin, and epigallocatechin gallate (EGCG), have been shown to alter epigenetic mechanisms. Some studies expected a beneficial outcome in using these phytochemicals to relieve the oxidative stress of diabetic patients [25]. For example, quercetin, an epi-drug present in citrus fruits and buckwheat, acts as a DNMT1 (deoxyribonucleic acid methyltransferase) inhibitor (via the repression of TNF-induced NF kappa transcription factor) and promotes Fas ligand related apoptosis via histone H3 acetylation and potential HDAC (histone deacetylase) inhibition. In addition, quercetin was found to stimulate glucose uptake through MAPK (mitogen-activated protein kinases) insulin-dependent mechanism. This is achieved in the liver through downregulation of gluconeogenesis enzymes and in the muscle through the translocation of GLUT4 (glucose transporters 4) (Figure 3) [25, 26].

The article "Anti-Diabesity Middle Eastern Medicinal Plants and Their Action Mechanisms" was published in 2022. Journal: Evid Based Complement Alternat Med.

Results obtained in animal studies and clinical trials confirm the traditionally known antidiabetic effects of several plants. These include pomegranate fruit, *Salvia*, *Trigonella foenum-graecum*, *Vaccinium arctostaphylos*, *Allium sativum*, *officinalis*, *Teucrium polium*, *Cinnamomum zeylanicum*, *Citrullus colocynthis*, *Urtica dioica*, and *Juglans regia*, not forgetting *black seeds* and *olive leaves/oil*. Furthermore, surveys carried out among healers of the Greco-Arabic and Islamic medicine in the Middle East revealed 26 new plants for the management of T2D. *Atriplex halimus L*. (salt bush)*, Cinnamomum zeylanicum* (Ceylon cinnamon), *Juglans regia L*. (walnut), *Ocimum tenuiflorum* (holy basil), *Olea europaea L*. (olive), *Trigonella foenum-graecum* (fenugreek), *and Urtica dioica L*. (nettle) are only a few of the medicinal plants that are strongly suggested (Table 1) as antidiabetics [25, 44, 53]. Fenugreek (*Trigonella foenum-graecum*) is a medicinal plant from Fabaceae family. A recent randomized, double-blind, placebo-controlled, clinical trial [58] has investigated the effects fenugreek as therapeutic complement for patients with borderline hyperlipidemia. Polyphenols have been proven in animal experiments to help reduce obesity and animal weight, as well as triglycerides, by boosting fat utilization and energy expenditure, as well as managing glucose homeostasis. Human research, on the other hand, has shown inconsistent results in terms of anti-obesity effectiveness. Variations in the results might be due to differences in the study subjects, trial design, length, and chemical forms. More examination of these factors (especially using randomized controlled trials) might lead to more clear findings on the medicinal potential of polyphenols obtained from herbs. The anti-hyperlipidemia effects of lemon balm (*Melissa officinalis*) were investigated in another recent randomized double-blind placebo-controlled clinical experiment [59]. The results of that study demonstrate that following supplementation, the mean LDL in the MO group was considerably lower than that in the placebo group. Although there was no significant change in cholesterol, FBG, HDL, triglyceride, creatinine, or ALT levels between the two groups after two months, there was a significant difference in AST levels. The findings showed that supplementation with *M. officinalis*, which is rich in antioxidants and bioactive compounds, can help lower LDL and AST levels in patients with borderline hyperlipidemia. Although numerous single herbs are experimentally or clinically reported to possess antidiabetic effects (Table 1), significantly less research has been directed to polyherbal mixtures. It is assumed that herbal products with various plant compounds have synergistic antidiabetic effects and will augment the specified actions. Several medicinal plant mixtures were evaluated for their antidiabetic effects. For instance, diasulin, a polyherbal mixture, contains both *Cassia auriculata* and *Gymnema sylvestre*, which can induce hypoglycemia by inhibiting intestinal glucose absorption and enhancing pancreatic insulin secretion, respectively. Additionally, the presence of *Trigonella foenum-graecum* during this mixture may decrease blood glucose by enhancing insulin secretion, increasing glucose uptake by tissues, decreasing intestinal glucose absorption, and inhibiting gluconeogenesis and glycogenolysis in hepatocytes. Diabetic dyslipidemia, which is often present in diabetic patients, is one of the main risk factors for CVDs. It is distinguished by an elevation in serum triglyceride and LDL cholesterol levels accompanied by a decrease in HDL cholesterol levels. The main objective of T2D dyslipidemia management is to lower serum LDL levels, which is well documented. Despite medication, the majority of T2D patients do not achieve the desired LDL values (<100 mg/dL) [60–63].

The article "Anti-Diabesity Middle Eastern Medicinal Plants and Their Action Mechanisms" was published in 2022. Journal: Evid Based Complement Alternat Med.

One of the commonly prescribed “antidiabetic” polyherbal mixtures by European herbalists is made of *Rubus fruticosus* and *Vaccinium myrtillus* leaves, *Potentilla erecta* roots, *Geum urbanum* aerial parts, and *Phaseolus vulgaris* pods. A recent study has evaluated the phytochemical composition; antioxidant capacity; potential toxicity; and hypoglycemic, hypolipidemic, nephroprotective, and hepatoprotective activities of this polyherbal mixture decoction. The results obtained in that study indicate that treatment with this mixture is more effective than the standard drugs (insulin and metformin) in the amelioration of hyperglycemia, hyperlipidemia, and histopathological changes of the pancreas, kidney, and liver tissue [63].

A plant mixture of water/ethanol extracts of *Juglans regia*, *Olea europaea* (leaves), *Urtica dioica* (aerial parts), and *Atriplex halimus* (leaves) is used in the traditional Greco-Arab and Islamic herbal medicine in the treatment of T2D. Increased glucose uptake by yeast cells, decreased glucose absorption in the rat intestine, and a substantial drop in blood glucose levels in streptozotocin-induced T2D rats were all used to illustrate the mixture's antidiabetic benefits. In 16 human volunteers with T2D, clinically acceptable glucose levels were achieved within 2-3 weeks of therapy. Within the first week, the plant mixture significantly reduced the glucose levels from 290 ± 40 to 210 ± 20 mg/dL. In addition, six patients treated with “Glucolevel” showed a substantial decrease in hemoglobin A1c levels. The action methods whereby the four plants employ their antidiabetic properties seem to be facilitated through synergistically different mechanisms that target glucose homeostasis. Scientific evidence obtained hitherto indicates hypoglycemic and antioxidant properties of each of the four used herbs. Oleuropein (the main active compound of *Olea europaea*) showed a distinct hypoglycemic effect at a dose of 16 mg/kg, together with hypotensive and hypolipidemic effects. Tannins and polyphenolics in *Juglans regia* leaves were found to be potent antioxidants and to reveal strong scavenging activity against free radicals. Extracts from *Atriplex halimus* and *Urtica dioica* were found to be effective in the treatment of T2D. Furthermore, they demonstrate insulin potentiating effects in animal models. “Glucolevel” enhances glucose access to yeast cells during anaerobic fermentation, which might be attributed to the presence of *Atriplex halimus* in the product, according to in vitro studies. The *Urtica dioica* component is hypothesized to lower glucose production in the liver, while oleuropein and tannins present in *Olea europaea* and *Juglans regia* leaves act as glucosidase inhibitors, restricting carbohydrate absorption in the intestine [64].

## 4. Herbal and Diet-Based Strategies to Prevent Diabesity-Related Hypertension

It is quite evident that environmental factors, as well as genetic and epigenetic mechanisms, play an important role in the development of hypertension. Obesity was found in various epidemiological studies to indicate one of the major causes of hypertension, which further highlights the fact that BMI and hypertension are almost linear within the general population. Several potential biochemical/molecular pathways are now known to contribute to the development of obesity-related hypertension [65, 66]. Several genes linked to diabetes, obesity, and hypertension have been revealed, and the number of obesity-associated genes is increasing day by day. In addition, activation of the renin-angiotensin-aldosterone system, hyperinsulinemia, elevated levels of cytokines acting at the endothelial cells, as well as abnormal levels of leptin, are also involved in the development of hypertension [36, 65, 66].

The article "Anti-Diabesity Middle Eastern Medicinal Plants and Their Action Mechanisms" was published in 2022. Journal: Evid Based Complement Alternat Med.

Recent clinical studies propose that excess of fat accumulation is not the principal inducer of the rise of obesity-related diseases, but the body fat distribution is a more significant factor for the disease. Generally, there are two forms of fat storage: visceral (intra-abdominal, surrounding internal organs) and subcutaneous (being stuck between skin and outer abdominal wall). Intra-abdominal fat and peripheral subcutaneous fat have distinct effects on the pathogenesis of obesity-related CVD. Visceral adiposity is connected with the development of hypertension, hyperlipidemia, T2D, and atherosclerosis. Visceral adipose tissue adipocytes and macrophages produce several proinflammatory cytokines but less anti-inflammatory mediators. Abnormal levels of these cytokines have significant contribution to the development of insulin resistance and play chief role in the pathogenesis of endothelium tissue and, as a response, atherosclerosis [65, 66].

It is widely documented that medicinal plants and nutritive changes play an important role in managing blood pressure. In highly motivated subjects, dietary changes are effective in lowering the blood pressure and in serving as initial treatment prior to drug therapy in uncomplicated stage-1 hypertension (with a systolic pressure ranging from 140 to 159 mm·Hg or a diastolic pressure ranging from 90 to 99 mm·Hg) [25, 36, 67–69].

Table 1 summarizes the commonly used antihypertensive medicinal plants. It is well documented that black seed (*Nigella sativa*) and Ginger *(Zingiber officinale)* have anti-diabesity effects and beneficial effects on diabetes-related diseases.

### 4.1. Black Seed (*Nigella sativa*)

The exact pathway of the hypotensive effects of black seed is not exactly elucidated. Potential pathways include synergistic effects of its active compounds, each with distinct molecular target and action mechanisms that result in a cardiac calming effect, calcium channels blocking property, and diuretic effects [70–72].

The article "Anti-Diabesity Middle Eastern Medicinal Plants and Their Action Mechanisms" was published in 2022. Journal: Evid Based Complement Alternat Med.

Regarding cardiac depressant effects, volatile oil and thymoquinone (the most abundant constituent of the volatile oil of *Nigella sativa* seeds) were found to lower both the arterial blood pressure and heart rate in animal test models. Cyproheptadine and atropine reversed these activities, indicating the contribution of serotoninergic and muscarinic receptors to the defensive properties of *Nigella sativa* [73, 74]. Furthermore, hexamethonium (a ganglionic blocker) prevented *Nigella sativa's* cardiac depressive effects in rats, revealing a nicotinic receptor route. Moreover, spinal pithing decreased *Nigella sativa*-induced cardiovascular effects by disrupting the link between the vasomotor core of the medulla and the preganglionic sympathetic neurons. As a result, the cardiac depressant and hypotensive actions of *Nigella sativa* appear to be mediated by a central mechanism involving a vasomotor center in the medulla and sympathetic output to the periphery [73, 74].

In respect of calcium channel blockade, thymol (one of the active compounds of *Nigella sativa*) has been found to target calcium (Ca^2+^) ion channels and hence lower blood pressure. It induced a dose-dependent relaxation in rat aorta. The Nigella sativa-derived active compounds caused endothelium-independent relaxation. This effect seems to be mediated through inhibition of Ca2+ release from sarcoplasmic reticulum, reduced Ca2+ sensitivity of the contractile system, and/or blockade of Ca2+ influx across the membrane. Thus, thymol caused a dose-dependent negative inotropic effect isolated cardiac preparation from canine and guinea pig. These activities seem to be the result of reduced Ca^2+^ levels in sarcoplasmic reticulum through blocking of the Ca^2+^ channel [73, 74].

Diuretic effects seem to be involved in the hypotensive effects of *Nigella sativa*. A decrease in water content and electrolyte concentrations declines blood volume and is one of the main mechanisms for control of the blood pressure. The diuretic effects of *Nigella sativa* were comparable to effects of 5 mg/kg of furosemide (a diuretic). An increase in urine excretion of Na^+^, K^+^, Cl, and urea causes these consequences. *Nigella sativa* extract was also shown to improve glomerular filtration rate, urine output, and electrolyte output. Blood pressure is controlled by the rennin-angiotensin-aldosterone system, which regulates blood volume and peripheral vascular resistance. However, 20 days of black seed therapy had no effect on the activities of plasma angiotensin-1-converting enzyme (ACE) and rennin in spontaneously hypertensive rats. As a result, *Nigella sativa's* hypotensive actions appear to be independent of the rennin-angiotensin-aldosterone system. However, further research is required to back up this assertion [25, 26, 36, 72–75].

The article "Anti-Diabesity Middle Eastern Medicinal Plants and Their Action Mechanisms" was published in 2022. Journal: Evid Based Complement Alternat Med.

### 4.2. Ginger (*Zingiber officinale*)

Ginger is one of the most broadly utilized herbs in traditional medicine for hypertension and CVD control and prevention. It lowers LDL and total cholesterol levels, which prevents the formation of sticky plaque along the walls of blood vessels and improves artery flexibility. *Zingiber officinale* and its active components (6-shogaol and 6-gingerol) target blood pressure and heart rate through direct and indirect mechanisms, according to several animal studies. Ginger crude extracts, for example, reduced arterial blood pressure in anesthetized rats in a dose-dependent manner, had a cardio-depressant effect on the pace and force of spontaneous contractions in guinea-pig paired atria, and relaxed phenylephrine-induced vascular contractions [36, 72, 74].

Calcium channel-blocking actions of *Zingiber officinale* crude extracts were seen when the crude extracts moved the calcium dose–response curves to the right, similar to the effect of verapamil. They also blocked the phenylephrine effect in both the absence and presence of calcium in the media. Hence, they target the plasma membrane-bound and intracellular calcium channels. Although L-NAME and atropine failed to suppress the vasodilator activity of *Zingiber officinale* crude extracts, they were found to be endothelium-independent. Hence, ginger's hypotensive actions are mediated via voltage-dependent calcium channel blockage. The hypotension-lowering effects of *Zingiber officinale* extract were aided in another study by the activation of both muscarinic receptors and calcium channel inhibition [36, 75, 76].

### 4.3. Artichoke (*Cynara scolymus*)

Artichoke, often known as globe artichoke, is an ancient perennial plant species native to the Mediterranean Basin, including North Africa and Southern Europe, and is now widely farmed all over the world. Because of its high abundance of bioactive phenolic components such as caffeoylquinic derivatives and flavonoids like apigenin and luteolin, the globe artichoke has a high nutritional value. Artichoke dried leaves and extracts have been utilized for antioxidant, choleretic, and pre- and probiotic activity, as well as hypoglycemic, hepatoprotective, cardiovascular health, and antiatherosclerotic properties, all of which are linked to flavonoid concentration [77]. In an 8-week double-blind, placebo-controlled, randomized experiment with an emphasis on volatile and nonvolatile chemicals, the effects of *Cynara scolymus* leaf powder on blood pressure and weight reduction in hypertensive patients as a supplemental treatment with Captopril were explored. The therapeutic effectiveness of *C. scolymus* as an adjuvant to Captopril on blood pressure and body mass index (BMI) in hypertensive individuals was investigated in that study. When comparing the *Cynara scolymus* group to the placebo group, there was a substantial improvement in BMI (*p*=0.04). The findings showed that consuming *Cynara scolymus* powder, which is high in phenolic and antioxidant chemicals, might help lower BMI and SBP in hypertensive individuals. Additional research is needed to validate or disprove the antihypertensive effect of artichoke [77].

The article "Anti-Diabesity Middle Eastern Medicinal Plants and Their Action Mechanisms" was published in 2022. Journal: Evid Based Complement Alternat Med.

### 4.4. Sumac (*Rhus coriaria* L., Anacardiaceae)

*Rhus coriaria* L., commonly called tanner's sumac, is a member of Anacardiaceae family. Sumac, which has traditionally been used to treat cardiovascular disorders, was shown to have positive benefits for CDV [78]. Sumac's hypotensive action was investigated in a randomized, double-blind, placebo-controlled clinical experiment [57, 78]. After 8 weeks, the *Rhus coriaria* L. group showed a substantial reduction in hypertension when compared to the baseline and placebo groups, but no significant change in BMI when compared to the baseline and placebo groups. Furthermore, the flavonoids luteolin, apigenin, and quercetin were shown to be the most abundant phenolic components in *Rhus coriaria* L. fruits. That research shows that the fruits of *Rhus coriaria* L. might be utilized as a natural treatment for hypertension. This plant's antihypertensive effect might be related to flavonoids, which were the plant's principal chemical ingredients [78].

## 5. Herbal and Diet-Based Strategies to Prevent Diabesity-Related Cardiovascular Disease

One of the best-explored diets for cardiovascular health is the traditional Mediterranean diet. It is well-known by its high content of vegetables, edible wild plants, nuts, fruits, grains, and olive oil. It has been found to lower the burden of CVD, hypertension, T2D, obesity, breast and colorectal cancers, asthma, and cognitive weakness [36]. It improves CVD indices, such as waist-to-hip ratio, lipid profile, and inflammatory mediators. These positive effects simply equal those seen with more conventional drugs used to treat CVD such as beta-blockers, aspirin, and angiotensin-converting enzyme inhibitors. However, it is undecided if this diet offers CVD advantage due to its separate components or due to additive and synergistic effects of its single components. Thanks to its antioxidant effects and hypotensive effects, the Mediterranean diet offers people a simple alternative to red meat-containing diet to achieve a lower incidence of CVD [79–81].

The article "Anti-Diabesity Middle Eastern Medicinal Plants and Their Action Mechanisms" was published in 2022. Journal: Evid Based Complement Alternat Med.

Olive oil and olive leaves are widely consumed in the traditional diets of most Mediterranean people. Apigenin, luteolin, oleuropein, verbascoside, and triterpenoids (oleanolic and maslinic acids) are the main active compounds in olive oil and its leaves (Figures 5 and 6). They contain monounsaturated fats, several antioxidant phenols, and other micronutrients that facilitate cardiovascular-protective effects. These include amelioration in oxidative stress, endothelial dysfunction, inflammation, thrombosis, blood pressure, and lipid and carbohydrate metabolism. Preventive effects on coronary heart disease were associated with high intake of olive oil and, above all, the extra-virgin type, which is rich in phenolic antioxidants. The cardioprotective effects were further supported by the results of a very recent analysis of two large US prospective cohort studies. Those studies show that higher olive oil consumption was connected to a lower risk of cardiovascular morbidity and mortality after 24 years of follow-up and that replacement of dairy fat, margarine, butter, or mayonnaise with the equivalent amount of olive oil significantly reduced CV risk [25, 36, 44, 82, 83].

The cholesterol-lowering action and the hypotensive effect of olive leaves are well acknowledged [81, 84]. A stable olive leaf extract (EFLA^®^ 943) has been pre-clinically tested for its antihypertensive effects as well as for its safety. For instance, in a preliminary clinical study carried out in 20 monozygotic adult twin pairs with mild hypertension in Germany, EFLA^®^ 943 (500 or 1,000 mg daily for 8 weeks) showed a significant reduction of patients' systolic blood pressure and diastolic blood pressure, compared to the control group. At a dose of 1 g/daily, the extract was clearly superior to recommendations for lifestyle changes in reducing mean blood pressure values from the baseline. The study also showed that at both doses the extract provided a significant reduction of LDL cholesterol level [81, 84]. Another double-blind, randomized, parallel and active-controlled clinical study evaluated the hypotensive effects as well as the tolerability of olive leaf extract in comparison with Captopril in patients with stage-1 hypertension [68]. It consisted of a run-in period of 4 weeks continued subsequently by an 8-week treatment period. EFLA^®^ 943 was given orally at the dose of 500 mg twice daily for 8 weeks. Captopril was given at the dosage regimen of 12.5 mg twice/day at start. The mean systolic blood pressure was 149.35.58 mm·Hg in the olive group and 148.45.56 mm·Hg in the Captopril group at baseline, according to the findings, while the mean diastolic blood pressure was 93.94.51 and 93.84.88 mm·Hg, respectively. Both groups exhibited a considerable drop in systolic and diastolic blood pressure from baseline after 8 weeks of therapy, with no significant differences between the groups. The olive and Captopril groups had mean systolic blood pressure reductions of 11.58.5 and 13.77.2 mm·Hg, respectively, and diastolic blood pressure reductions of 4.85.5 and 6.45.2 mm·Hg, respectively, from baseline to the conclusion of the research. The olive group, but not the Captopril group, showed a considerable reduction in triglyceride levels [68].

The article "Anti-Diabesity Middle Eastern Medicinal Plants and Their Action Mechanisms" was published in 2022. Journal: Evid Based Complement Alternat Med.

Many prospective studies confirmed the cardiovascular values of diets with olive oil as main ingredient. Most of these reports were conducted in the Mediterranean Basin. For instance, the connection between olive oil consumption and all-cause as well as cause-specific mortality was studied in a Spanish population. A significant decline in CVD mortality is connected with continuing increased dietary intake of olive oil [36, 79–81, 84–86]. The relation between the amount of olive oil consumption and the incidence of coronary heart disease was evaluated in two prospective studies. In a Spanish cohort study, people who consumed more than 28.9 g of olive oil per day had a slightly lower risk of coronary heart disease (−22%). In a three-city study in France, individuals who consumed olive oil intensively had a 41% less risk of stroke than those who did not [79–81, 84–87]. Another multicenter trial in Spain was conducted among participants (men being 55 to 80 years of age and women being 60 to 80 years of age) with no CVD at enrolment, though at high cardiovascular risk. They had either T2D or at least three of the following risk factors: hypertension, smoking, low HDL levels, high LDL levels, overweight/obesity, or a family history of coronary heart disease. The patients were asked to consume one of the following diets: A Mediterranean diet enriched either with extra-virgin olive oil or with mixed nuts. The control group was adviced to reduce dietary fat. Myocardial infarction, stroke, and death from cardiovascular causes were the chief end endpoints. The test was ended after a median follow-up of 4.8 years, based on the results of an interim analysis. According to the findings of such a multicenter primary prevention trial, an energy-unrestricted Mediterranean diet supplemented with extra-virgin olive oil or nuts resulted in significant reduction in the incidence of major cardiovascular events among high-risk adults. The findings back up the Mediterranean diet's long-held reputation for lowering the risk of cardiovascular disease [36, 79–81, 84–87].

The article "Anti-Diabesity Middle Eastern Medicinal Plants and Their Action Mechanisms" was published in 2022. Journal: Evid Based Complement Alternat Med.

Regular consumption of vegetables and fruits is suggested practically by every Mediterranean diet. The WHO recommends the dietary intake of a minimum of 400 g of fruits and vegetables per day [83]. According to a recent meta-analysis, consuming 800 g of fruit per day was linked to a 27% reduction in the relative risk of CVD [84]. Following multivariate normalization, epidemiological data revealed substantial inverted correlations between flavonoid-rich fruit (e.g., strawberries, grapefruit) and coronary heart disease mortality in CVD-free postmenopausal women [88, 89]. Intervention trials provided evidence that consumption of a variety of fruits and fruit juices has also been shown to lessen cardiovascular dysfunction risk factors. For example, endothelial dysfunction, dyslipidemia, platelet aggregation, and hypertension have all been shown to be improved by consuming fruit high in anthocyanins and procyanidins, such as berries [90], while flavanone-rich citrus, such as orange, has been shown to improve hypercholesterolemia [7]. The intake of cherries was found to promote cardiovascular health by hypolipidemic and anti-inflammation effects [91]. According to an epidemiological research, drinking fruit juice, such as citrus, berries, and cherry juice, has also been shown to improve vascular health by lowering risk factors such as blood pressure and lipid profiles [92]. Remarkably, the potential benefit of fruits and vegetables could lie in decreased total caloric burden or in the synergistic activities of many active compounds, nutrients, and vitamins that they offer. Significant antioxidant properties of fruits and vegetables, as well as the health benefits of increased intake of plant polyphenols (strong antioxidants) and concomitant weight loss associated with diets high in fruits and vegetables, are the main mechanisms by which they exert their beneficial cardiovascular effects [80].

A number of observational analyses in the Mediterranean region uncovered that fruit and vegetable consumption is inversely connected with blood pressure, BMI, and fatal ischemic heart disease. For example, in a 2004 cross-sectional analysis of a prospective cohort study, fruit and vegetable consumption was found to be negatively related to blood pressure in a Mediterranean community with a high vegetable-fat intake. Additional cross-sectional analysis showed that augmented fruit and vegetable intake is related to a reduced BMI. Although the results were significantly biased by heterogeneity and publication bias, a major 2006 meta-analysis of over 200,000 patients indicated a 4% relative risk reduction in CVD with each serving of vegetables and a 7% relative risk reduction in CVD with each daily increase in servings of fruit. Another major meta-analysis of observational trials (almost 200,000 patients) found that eating 3–5 servings of fruits and vegetables per day reduced CVD occurrences by 17%. After an eight-year follow-up of 313,074 patients without atherosclerosis, population-based evidence from the European prospective investigation into cancer and nutrition study revealed that those who ate eight portions of fruits and vegetables per day had a 22% lower risk of fatal ischemic heart disease than those who ate three portions or less [93, 94].

The article "Anti-Diabesity Middle Eastern Medicinal Plants and Their Action Mechanisms" was published in 2022. Journal: Evid Based Complement Alternat Med.

Tomatoes should be consumed on a regular basis as part of any Mediterranean diet. Lycopene is the principal carotenoid found in tomato-based goods, and it has been linked to a reduced risk of cancer, cardiovascular disease, cognitive impairment, and osteoporosis. Tomatoes in the diet increase the body's antioxidant levels, trapping reactive oxygen species and minimizing oxidative damage to essential macromolecules including membrane lipids, enzyme proteins, and DNA, lowering oxidative stress. As a result, they are useful in protecting the human body from various diseases caused by oxidative stress. The most frequent phenolic chemicals found in tomatoes are quercetin, kaempferol, naringenin, caffeic acid, and lutein [95].

A recent clinical trial was conducted on 150 healthy subjects who consumed tomato-based product (Cardi-O-Mato) or placebo for two weeks. The test group had significantly lower levels of oxidized LDL and lower insulin levels compared to the placebo group. Moreover, a beneficial trend was also observed for post-meal glucose levels [96].

Several reports of epidemiological studies have appeared in support of the traditionally known benefits of lycopene in the avoidance of CVD. Antioxidant scavenger and inhibition of proinflammatory and pro-thrombotic mediators are the main contributors of the reported lycopene benefits in CVD prevention. Although many features of lycopene *in vivo* metabolism, functions, and clinical indications remain to be explained, lycopene at low doses has been reported to be a preventive measure for ameliorating various aspects of CVD [97, 98]. A recent systematic review and meta-analysis on the effect of supplementing tomato and lycopene on cardiovascular risk factors has supported the opinion that increasing the intake of these has ameliorating effects on blood pressure and endothelial function [99].

Due to the widespread availability of refined grains and the relevance of the gut flora, dietary fibers have recently been a focus of scientific studies. Dietary fibers from beans, fruits, and vegetables were correlated to the composition of the gut microbiome in a human study. Obesity and related disorders, such as metabolic syndrome, have been linked to these microbiome alterations. In terms of high fiber consumption and health outcomes, it has been associated with beneficial effects on cardiovascular risk factors including hypertension and hyperlipidemia. Despite the insufficient data in cohort trials, a meta-analysis found an inverse relationship between dietary fiber consumption and metabolic syndrome in cross-sectional studies but not in cohort studies [100].

The article "Anti-Diabesity Middle Eastern Medicinal Plants and Their Action Mechanisms" was published in 2022. Journal: Evid Based Complement Alternat Med.

Several lines of epidemiological evidence prove a contrary association between augmented food fiber consumption (e.g., cereal fiber, fruit, vegetables) and CVD risk. The connection has been found to be significantly higher with cereal fiber compared to fruit or vegetable fiber. Numerous studies have also shown increased whole grain intake to be associated with CVD risk reduction. Based on these indications, recent US dietary strategies have suggested the daily consumption of 25–30 g of fiber rich whole grains. Regular intake of cereal dietary fiber supports cardiovascular health through multiple mechanisms. According to several observational studies, benefits were mediated through improving glucose metabolism (lower absorption of lipids and simple carbohydrates), antioxidant effects, blood pressure regulation, inflammation reduction, lipid reduction, and weight loss [36, 93, 94].

A number of observational reports prove that nut intake is linked with a reduced risk of T2D, coronary artery disease, and hypertension [32, 80, 101, 102]. It decreases CVD risk factors, including amendments in triglycerides, total cholesterol, and LDL cholesterol levels [101]. As previously mentioned, several randomized control trials linked a nut-rich Mediterranean diet to lower risk of CVD. A substantial number of cohort studies and quite a few smaller randomized control trials suggest that the observed amendment of cardiovascular morbidity and mortality is the result of a decrease in lipid profiles and reactive oxygen species as well as hypotensive effects. Additionally, such definitive results concerning the effect of daily nut intake on CVD prevention would certainly attribute it to being a diet that can be followed on its own, without the added advantage of the Mediterranean diet, although nut consumption can give higher CVD benefit when combined with the Mediterranean diet [80, 102].

Almonds are approved by the FDA thanks to their beneficial effects in lowering CVD risks. They are rich in dietary fiber, vitamin E, and monounsaturated fats. Almond consumption was found to reduce the levels of LDL cholesterol, but it does not affect HDL as reported in a meta-analysis of lipid-neutralising potential conducted on normolipidemic, prediabetic and/or diabetic, obese, and/or hyperlipidemic persons [69, 84–86]. A randomized controlled trial conducted on coronary artery disease (CAD) patients has found that dietary almonds increase serum HDL cholesterol [102]. Even with normal LDL levels in CAD patients, reduced HDL levels represent an independent indicator of CVD risk. Almost 50% of CAD's hospitalized patients have normal LDL cholesterol but low HDL levels. The effect of almonds on HDL cholesterol in CAD patients starting with low HDL cholesterol was evaluated in another randomized controlled clinical trial [103]. According to the findings of that study, almonds dramatically increase HDL levels. HDL values were 12–16% higher at weeks 6 and 12 compared to the corresponding baseline. Total cholesterol, triglycerides, LDL and VLDL serum levels, total-to-HDL and LDL-to-HDL ratios, and atherogenic index were all decreased at weeks 6 and 12 compared to baseline, confirming prior findings. Eventually, daily intake of 10 g almonds before breakfast can improve HDL levels while also enhancing other lipid profile markers in CAD patients with low HDL cholesterol [80, 103–105].

The article "Anti-Diabesity Middle Eastern Medicinal Plants and Their Action Mechanisms" was published in 2022. Journal: Evid Based Complement Alternat Med.

Two large cohorts of US studies tested the relationship between regular nut intake and inflammatory biomarkers in 5,013 subjects who were free of diabetes. Nut intake (e.g., peanuts and other nuts) was estimated from food-frequency questionnaires and from cumulative averages from 1986 to 1990 in the Nurses' Health Study (NHS) and from 1990 to 1994 in the Health Professionals Follow-Up Study (HPFS). Plasma samples were collected in the NHS in 1989–1990 and the HPFS in 1993–1995. Regular nut eating was linked to a favorable inflammatory biomarker profile. Proinflammatory indicators such as C-reactive protein, IL-6, and TNF-receptor 2 were found to be in lower quantities [104].

Over the last few decades, several health benefits have been ascribed to polyphenols, and their pharmacological action mechanisms have been elucidated at biochemical and cell biological levels. These embrace, but are not limited to, anti-inflammatory, antioxidant, anticancer, antibacterial, antifungal, photo-protective, and protective activities against stress-induced disorders such as aging, rheumatoid arthritis, T2D, and cardiovascular and neurodegenerative diseases. Polyphenols comprise a large group of heterogeneous secondary metabolites found to be almost prevalent in the plant kingdom and act as primary defense mechanisms (phytoalexins) against different environmental stressors and pathological aggression [105–108].

The article "Anti-Diabesity Middle Eastern Medicinal Plants and Their Action Mechanisms" was published in 2022. Journal: Evid Based Complement Alternat Med.

Polyphenols are divided into two classes based on their chemical structures: flavonoids and non-flavonoid polyphenols, which include phenolic acids. They are most commonly found in combination with sugars or acylated sugars (glycosides), but they can also be found in other conjugated structures (amides, esters, and methyl ethers) or in their free form. Flavonoids are a kind of polyphenol that includes about 6,000 different chemicals. Flavonoids are classified as flavones, flavonols, flavanones, flavanonols, flavan-3-ols, anthocyanins, and isoflavones based on their hydroxylation and substitution patterns, as well as the degree of saturation of the chromane ring. Condensed tannins are polymers of flavan-3-ols or flavan-3,4-diols, sometimes known as proanthocyanidins or polyflavonoid tannins [105–107]. Non-flavonoid polyphenols have a more complex structure and include hydrolysable tannins (gallotannins and ellagitannins), lignans, stilbenes, and phenolic acids. The majority of phenolic acids found in food are benzoic acid or cinnamic acid derivatives [105–107].

According to evidence gathered from several epidemiological research works, eating polyphenol-rich fruits and vegetables lowers the risk of cancer and cardiovascular disease. A vast number of in vitro and animal experiments utilizing pure polyphenols backed up these findings [107, 108]. However, animal and clinical investigations have revealed that polyphenols have restricted absorption and a high hepatic metabolism, raising doubts about the validity of in vitro and animal studies on polyphenols [107, 108].

## 6. Herbal-Based Strategies to Prevent Diabetes-Related Nephropathy

T2D-related renal disease is characterized by functional as well as structural irregularities of the kidney. The most common cause of end-stage renal disease is diabetic nephropathy, which accounts for substantial morbidity and mortality. Kidney pathophysiology in diabetes is advanced by interactions between metabolic and haemodynamic factors. The changes may result from the effects of excess glucose directly on kidney cells or indirectly through pathways that involve development of oxidants and advanced glycation end-products [109–111]. Chronic hyperglycemia accelerates the activation of the formation of advanced glycation end-products (AGEs), polyol pathway, and protein kinase C pathway [110–114].

Current conventional T2D management using blood hypoglycemic drugs has limitations in avoiding the development of renal diseases. The start of T2D nephropathy is connected with a progressive rate of deterioration in renal function, urinary albumin excretion, and glomerular filtration rate (GFR). T2D treatment should therefore aim to intervene on promoters of the decline in renal function in diabetes to avert adverse consequences.

The article "Anti-Diabesity Middle Eastern Medicinal Plants and Their Action Mechanisms" was published in 2022. Journal: Evid Based Complement Alternat Med.

Accumulative indication suggests that some herbal extracts with hypoglycemic properties may have beneficial effects on some processes associated with a decline in renal function, as well as reducing the severity of nephropathy in T2D experimental animals. Table 1 summarizes the most commonly used anti-nephropathy herbals [114]. Based on various experimental studies, traditional medicinal plants and their bioactive constituents control the cellular processes involved in the initiation of nephropathy owing to their significant pharmacological activities; however, their efficacy has not yet been explored in animal test models and in clinical studies. Consequently, studies must be done to assess the nephroprotective effects of medicinal plants in preclinical animal models and in humans. Medicinal plants have various bioactive constituents, which may slow the progression of nephropathy and improve renal function through targeting multiple pathways, including p38MAPK (p38 mitogen-activated protein kinases), JNK (c-Jun N-terminal kinases), transforming growth factor beta (TGF-*β*), NF-*κ*B (nuclear factor kappa-light-chain-enhancer of activated B cells), Wnt, and JAK-STAT signaling pathway. Depletion or inhibition of these accelerating factors may provide a significant therapy for nephropathy [115–118].

## 7. Concluding Remarks

The current strategy in diabesity management is targeting enzymes that regulate carbohydrate and lipid metabolism. Side effects produced by pharmaceutical anti-diabesity drugs have obliged the search for new novel drugs. In recent years, medicinal plants and phytochemicals have had importance for the management of both obesity and diabetes. Their synergistic and multi-targeted effects represent a promising alternative in the management of diabesity. Some phytochemicals regulate gene expression involved in metabolic pathways like adiponectin gene expression and peroxisome proliferator-activated receptor gamma. In addition, they are able to inhibit metabolic enzymes like lipases, amylases, and glucosidases. Medicinal plants present a spring of natural multifunctional molecules. Many phytochemicals including flavonoids have been reported for multi-functionality. The chemical structure of flavonoids affects the activity of lipases and glucosidases, which can be valuable for development of new anti-diabesity drugs.

The further acceptance of herbal and diet-based remedies needs to be supported by large clinical studies including studies on toxicity and bioavailability. The Mediterranean diet, based on the traditional diet of many North African and Southern European as well as Middle Eastern countries, contains proportionally high quantities of olive oil, legumes, unrefined cereals, vegetables, and fruits. It also includes moderate consumption of dairy products (mostly cheese and yogurt) and wine, low consumption of meat and meat products, and adequate to high consumption of fish. However, this diet is being followed by many people worldwide as a part of a healthy lifestyle. Based on what has been explored herein, the Mediterranean diet provides suitable quantities of a diversity of antioxidants, including known vitamins or phytochemicals. The Mediterranean diet with extra-virgin olive oil or nuts was found to lessen the incidence of major cardiovascular diseases. An inverse association between adherence to the Mediterranean diet and cardiovascular risk was reported in observational cohort studies and a secondary prevention trial. The Mediterranean diet's hypotensive effects are believed to be mediated by antioxidants, cardiac depressants, diuretics, and calcium channel blockage [36–39, 44, 50–52, 119]. The majority of published evidence, on the other hand, comes from animal trials or cell culture platforms. Hence, clinical trials to assess the effectiveness and safety of herbal-based therapies are important.

The article "Anti-Diabesity Middle Eastern Medicinal Plants and Their Action Mechanisms" was published in 2022. Journal: Evid Based Complement Alternat Med.

## Figures and Tables

**Figure 1:** The interconnection between obesity and T2D.

**Figure 2:** Main classes of herbal secondary metabolites, their herbal sources, and their anti-obesity activities.

**Figure 3:** Anti-diabesity action mechanisms of medicinal plants.

**Figure 4:** Potential synergistic anti-diabesity molecular multiple targets of diet- and medicinal herbal secondary metabolites. NOS: nitric oxide synthase; ROS : reactive oxygen species; TLR4 : Toll-like receptor 4; MCP-1 : monocyte chemoattractant protein-1; PPAR*γ* : peroxisome proliferator-activated receptor gamma; NF-*κ*B : nuclear factor-*κ*B; TNF-*α* : tumor necrosis factor alpha.

**Figure 5:** Anti-diabesity effects of *Olea europaea*. COX: cyclooxygenase; GSH: reduced glutathione; GST: glutathione-S-transferase; IFN-*γ*: interferon gamma; IL: interleukine; iNOS: inducible nitric oxide synthase; LDL: low density lipoprotein; SOD: superoxide dismutase; TNF-*α*: tumor necrosis alpha.

**Figure 6:** Cardiovascular beneficial effects of the traditional Mediterranean diet. This diet is characterized by a high intake of olive oil, vegetables, nuts, fruits, and grains; a moderate intake of fish; and a low intake of red meat or processed meat. Beneficial cardiovascular activities are mediated through reduction of the blood pressure, improvement of lipid profile, reduction of oxidative stress, and weight loss.

The article "Anti-Diabesity Middle Eastern Medicinal Plants and Their Action Mechanisms" was published in 2022. Journal: Evid Based Complement Alternat Med.

**Table 1:** Commonly used medicinal plants in the treatment of obesity, diabetes, hypertension, cardiovascular disease, and nephropathy.

Plant name	Obesity	Diabetes	Hypertension	Cardiovascular disease	Nephropathy
*Acacia ligulata*	—	√	—	—	—
*Adonis palaestina*	√		√	√	
*Aegle marmelos*	√	√	—	√	—
*Aframomum melegueta*	√	—	—	—	—
*Allium sativum*	*√*	*√*	*√*	*√*	*√*
*Aloe vera*	—	√	—	—	—
*Alpinia zerumbet*	√	√	√	—	—
*Anchusa azurea*	√	—	—	—	—
*Arachis hypogaea*	—	—	√	—	√
*Aralia elata*	√	√	—	√	—
*Asparagus acutifolius*	√	—	—	—	—
*Bacopa monnieri*		—	—	—	√
*Bergenia crassifolia*	√	√	—	—	—
*Beyeria leschenaultii*		√	—	—	—
*Camellia sinensis*	√	√		√	√
*Capsicum annuum*	√	√	—	√	—
*Carthamus oxyacantha*	√	√	—	—	—
*Carthamus tinctorius*		√	—	√	—
*Cassia angustifolia*	√	√	—	—	—
*Castanea crenata*	√	—	—	—	—
*Catharanthus roseus*	—	√	√	√	
*Caulis polygoni*	√	√	—	—	—
*Cichorium intybus*	√	√	—	√	—
*Cynara scolymus*	√	√	√	√	√
*Cinnamomum zeylanicum*	√	√	—	√	—
*Citrus aurantium*	√	—	√	√	—
*Coffea arabica*	√	—	—	√	√
*Coleus forskohlii*	√	—	√	√	√
*Coptis chinensis*	√	√	—	—	√
*Corni fructus*	√		√	—	√
*Cornus officinalis*	√	√	—	√	√
*Cinnamomi ramulus*	√	—	√	—	—
*Costus pictus*	—	√	—	—	√
*Curcuma longa*	√	√	—	√	√
*Cynometra cauliflora*	√	√	—	—	—
*Dioscorea nipponica*	√	—	—	√	—
*Diplotaxis tenuifolia*	√	—	—	√	√
*Eleusine indica*	√	—	—	—	√
*Ephedra species*	√	—	√	√	—
*Eucalyptus galbie*	√	—	—	—	—
*Eugenia cumini*	—	√	√	—	—
*Eugenia polyantha*	—	√	√	—	—
*Euonymus alatus*	√	√	—	—	—
*Fagonia arabica*	√	—	—	—	—
*Fagonia cretica*	—	√	—	—	—
*Ferula asafoetida*	√	√	√	—	—
*Ficus carica*	√	√	—	√	—
*Foeniculum vulgare*	√	√	—	—	—
Fructus Amomi	√	√	—	—	√
*Garcinia cambogia*	√	√	—	—	—
*Geranium nepalense*	√	√	—	—	—
*Ginkgo biloba*	√	√	——	√	—
*Glycine max*	√	√	√	√	—
*Glycyrrhiza glabra*	—	√		—	—
*Gynostemma pentaphyllum*	—	√	—	—	—
*Helichrysum ceres*	—	—	√	√	√
*Hoodia gordonii*	√	√	√	—	—
*Hoodia pilifera*	√		—	—	—
*Humulus lupulus*	√	√	—	—	—
*Hypericum perforatum*	√	√	—	√	—
*Hypoxis hemerocallidea*	—	√	—	√	√
*Iostephane heterophylla*	—	√	—	—	—
*Juglans regia*	√	√	—	—	—
*Juniperus oxycedrus*	√	√	√	—	—
*Linum usitatissimum*	√	√	√	—	—
*Ludwigia octovalvis*	—	√	√	—	—
*Malva parviflora*	√	√	√	√	—
*Mangifera indica*	√	√	—	√	√
*Marrubium radiatum*	√	√	—	—	—
*Melastoma candidum*	√	—	—	√	—
*Melissa officinalis*	√	√	√	√	
*Mentha spicata*	√	√	√	—	—
*Millettia reticulata*	√	—	—	—	—
*Momordica charantia*	—	√	—	—	√
*Momordica charantia,*	√	√	√	—	√
*Moringa stenopetala*	√	√	√	—	—
*Morus alba*	√	√	√	√	—
*Mucuna pruriens*	—	√	√	—	√
*Myristica fragrans*	√	√	—	—	—
*Myrtus communis*	√	√	—	√	—
*Nelumbo nucifera*	√	√	—	√	
*Nigella sativa*	√	√	√	√	√
*Ocimum tenuiflorum*	—	√	√	√	—
*Olea europaea*	—	√	√	√	√
*Ononis natrix*	√	√	—	—	—
*Opuntia monacantha*	—	√	—	—	√
*Origanum syriaca*	√	—	—	—	√
*Origanum vulgare*	√	√	—	—	—
*Orixa japonica*	√	√	—	—	—
*Panax ginseng*	√	√	√	—	—
*Papaver rhoeas*	√	—	—	√	√
*Paronychia argentea*	√	—	—	—	√
*Passiflora nitida*	√	√	—	—	—
*Persea americana*	√	—	√	√	√
*Phaseolus vulgaris*	√	√		√	—
*Phyla nodiflora*	√	√	√		√
*Pimpinella anisum*	√	√	√	√	√
*Pinus koraiensis*	√	√	—	—	—
*Pistacia vera*	√	√	—	√	—
*Portulaca oleracea*	√	√	—	—	—
*Psidium guajava*	—	√	√	√	—
*Pterocarpus marsupium*	—	√	—	√	—
*Pyrus pyrifolia*	√	√			
*Raphanus raphanistrum*	√	—	√	√	√
*Rehmannia glutinosa*	√	√	√	—	—
*Reseda alba*	√	—	—	—	—
*Rheum emodi*	—	√	—	—	√
Rhizoma Alpiniae	—	√	—	—	√
Rhizoma Fagopyri	—	√	√	—	—
*Rhus coriaria*	√	√	√	√	
*Robinia pseudoacacia*	√	—	—	—	—
*Rosa damascena*	√	√		√	—
*Rosa rugosa*	√	√	√	—	—
*Rosmarinus officinalis*	√	√	√	√	√
*Rubi fructus*	√	√	√	—	—
Salicis Radicis	√	—	—	—	—
*Salvia acetabulosa*	—	√	—	—	—
*Salvia miltiorrhiza*	√	—	—	√	—
*Salvia spinosa*	√	—	—	—	—
*Santalum spicatum*	√	√	√	—	—
*Sclerocarya birrea*	—	√	√		√
*Shorea roxburghii*	√	√	√	√	
*Silybum marianum*	—	√	√	√	√
*Smilax glabra*	—	√	—	√	√
*Smyrnium olusatrum*	√	—	√		
*Sonchus asper*	√	√	√	—	√
*Sonchus oleraceus*	√	√	—	√	√
*Spilanthes acmella*	√	—	√	—	—
*Terminalia arjuna*	—	√	√	√	
*Trigonella foenum-graecum*	√	√	—	√	√
*Urtica urens*	√	√	—	—	—
*Vigna angularis*	√	√	√		√
*Vitis vinifera*	√	√	—	√	
*Zingiber officinale*	√	√	√	√	√

The article "Anti-Diabesity Middle Eastern Medicinal Plants and Their Action Mechanisms" was published in 2022. Journal: Evid Based Complement Alternat Med.

## Data Availability

The data used to support the findings of this study are available from the corresponding author upon request.

## References

[1] Rathod P., Yadav R. P. (2021). Anti-diabesity potential of various multifunctional natural molecules. *Journal of Herbal Medicine*.

[2] Safaei M., Sundararajan E. A., Driss M., Boulila W., Shapi’i A. (2021). A systematic literature review on obesity: understanding the causes & consequences of obesity and reviewing various machine learning approaches used to predict obesity. *Computers in Biology and Medicine*.

[3] Zhao X., He Q., Zeng Y., Cheng L. (2021). Effectiveness of combined exercise in people with type 2 diabetes and concurrent overweight/obesity: a systematic review and meta-analysis. *BMJ Open*.

[4] Field A. E., Coakley E. H., Must A. (2001). Impact of overweight on the risk of developing common chronic diseases during a 10-year period. *Archives of Internal Medicine*.

[5] Hart C. L., Hole D. J., Lawlor D. A., Davey Smith G. (2007). How many cases of type 2 diabetes mellitus are due to being overweight in middle age? Evidence from the Midspan prospective cohort studies using mention of diabetes mellitus on hospital discharge or death records. *Diabetic Medicine*.

The article "Anti-Diabesity Middle Eastern Medicinal Plants and Their Action Mechanisms" was published in 2022. Journal: Evid Based Complement Alternat Med.

[6] Narayan K. M., Boyle J. P., Thompson T. J., Gregg E. W., Williamson D. F. (2007). Effect of BMI on lifetime risk for diabetes in the U.S. *Diabetes Care*.

[7] Wannamethee S. G., Shaper A. G., Walker M. (2005). Overweight and obesity and weight change in middle aged men: impact on cardiovascular disease and diabetes. *Journal of Epidemiology & Community Health*.

[8] Montague C. T., O’Rahilly S. (2000). The perils of portliness: causes and consequences of visceral adiposity. *Diabetes*.

[9] Badran M., Laher I. (2011). Obesity in Arabic-speaking countries. *Journal of Obesity*.

[10] Hossain P., Kawar B., El Nahas M. (2007). Obesity and diabetes in the developing world—a growing challenge. *New England Journal of Medicine*.

[11] Ferraro K. F., Su Y. P., Gretebeck R. J., Black D. R., Badylak S. F. (2002). Body mass index and disability in adulthood: a 20-year panel study. *American Journal of Public Health*.

[12] Ramadan S., Ibrahim A. A. (2021). Fruits and vegetables as sources of functional phytochemicals for the prevention and management of obesity, diabetes, and cancer. *Dietary Phytochemicals*.

[13] Wild S. H., Roglic G., Green A., Sicree R., King H. (2004). Global prevalence of diabetes: estimates for the year 2000 and projections for 2030. *Diabetes Care*.

[14] Atlas Diabetes (2011). International diabetes federation. *IDF Diabetes Atlas*.

[15] Radwan H., Hasan H., Hamadeh R. (2020). Complementary and alternative medicine use among patients with type 2 diabetes living in the United Arab Emirates. *BMC Complement Med Ther*.

[16] Mokdad A. H., Ford E. S., Bowman B. A. (2003). Prevalence of obesity, diabetes, and obesity-related health risk factors. *JAMA*.

[17] Archer E., Lavie C. J. (2022). Obesity subtyping: the etiology, prevention, and management of acquired versus inherited obese phenotypes. *Nutrients*.

[18] Kiess W., Galler A., Reich A. (2001). Clinical aspects of obesity in childhood and adolescence. *Obesity Reviews*.

[19] Samama P., Rumennik L., Grippo J. F. (2003). The melanocortin receptor MCR4 controls fat consumption. *Regulatory Peptides*.

[20] Kurokawa N., Nakai K., Kameo S., Liu Z. M., Satoh H. (2001). Association of BMI with the *β*3-adrenergic receptor gene polymorphism in Japanese: meta-analysis. *Obesity Research*.

[21] Widen E., Lehto M., Kanninen T., Walston J., Shuldiner A. R., Groop L. C. (1995). Association of a polymorphism in the beta 3-adrenergic-receptor gene with features of the insulin resistance syndrome in Finns. *New England Journal of Medicine*.

[22] Halberg N., Henriksen M., Soderhamn N. (2005). Effect of intermittent fasting and refeeding on insulin action in healthy men. *Journal of Applied Physiology*.

The article "Anti-Diabesity Middle Eastern Medicinal Plants and Their Action Mechanisms" was published in 2022. Journal: Evid Based Complement Alternat Med.

[23] Burgio E., Lopomo A., Migliore L. (2015). Obesity and diabetes: from genetics to epigenetics. *Molecular Biology Reports*.

[24] Speakman J. R. (2006). Thrifty genes for obesity and the metabolic syndrome–time to call off the search?. *Diabetes and Vascular Disease Research*.

[25] Shanak S., Saad B., Zaid H. (2019). Metabolic and epigenetic action mechanisms of antidiabetic medicinal plants. *Evidence-Based Complementary and Alternative Medicine*.

[26] Saad B., Ghareeb B., Kmail A. (2021). Metabolic and epigenetics action mechanisms of antiobesity medicinal plants and phytochemicals. *Evidence-based Complementary and Alternative Medicine*.

[27] Bays H., Mandarino L., DeFronzo R. A. (2004). Role of the adipocyte, free fatty acids, and ectopic fat in pathogenesis of type 2 diabetes mellitus: peroxisomal proliferator-activated receptor agonists provide a rational therapeutic approach. *Journal of Clinical Endocrinology and Metabolism*.

[28] McGarry J. D. (2002). Banting lecture 2001: dysregulation of fatty acid metabolism in the etiology of type 2 diabetes. *Diabetes*.

[29] Roden M. (2005). Muscle triglycerides and mitochondrial function: possible mechanisms for the development of type 2 diabetes. *International Journal of Obesity*.

[30] Donath M. Y., Ehses J. A., Maedler K. (2005). Mechanisms of beta-cell death in type 2 diabetes. *Diabetes*.

[31] Abbasi F., Chu J. W., Lamendola C. (2004). Discrimination between obesity and insulin resistance in the relationship with adiponectin. *Diabetes*.

[32] Chen B. H., Song Y., Ding E. L. (2009). Circulating levels of resistin and risk of type 2 diabetes in men and women: results from two prospective cohorts. *Diabetes Care*.

[33] Knowler W. C., Barrett-Connor E., Fowler S. E. (2002). Reduction in the incidence of type 2 diabetes with lifestyle intervention or metformin. *New England Journal of Medicine*.

[34] Dunning B. E., Gerich J. E. (2007). The role of alpha-cell dysregulation in fasting and postprandial hyperglycemia in type 2 diabetes and therapeutic implications. *Endocrine Reviews*.

[35] Pratley R. (2006). Islet dysfunction: an underlying defect in the pathophysiology of type 2 diabetes. *Endocrinology and Metabolism Clinics of North America*.

[36] Saad B. (2019). Prevention and treatment of obesity-related cardiovascular diseases by diet and medicinal plants. *Herbal Medicine: Back to the Future*.

[37] Saad B., Said O. (2011). *Greco-Arab and Islamic Herbal Medicine: Traditional System, Ethics, Safety, Efficacy and Regulatory Issues*.

[38] Saad B., Azaizeh H., Abu Hijleh G., Said O. (2006). Safety of traditional Arab herbal medicine. *Evidence-based Complementary and Alternative Medicine*.

The article "Anti-Diabesity Middle Eastern Medicinal Plants and Their Action Mechanisms" was published in 2022. Journal: Evid Based Complement Alternat Med.

[39] Saad B. (2015). Integrating traditional Greco-Arab and Islamic herbal medicine in research and clinical practice. *Phytotherapies: Safety, Efficacy, and regulation*.

[40] Said O., Saad B., Fulder S., Khalil K., Kassis E. (2011). Weight loss in animals and humans treated with “weighlevel,” a combination of four medicinal plants used in traditional Arabic and islamic medicine. *Evidence-based Complementary and Alternative Medicine*.

[41] Saad B., Zaid H., Said O. (2013). Tradition and perspectives of diabetes treatment in greco-arab and islamic medicine. *Bioactive Food As Dietary Interventions For Diabetes*.

[42] Mohamed G. A., Ibrahim S. R., Elkhayat E. S., Salah El Dine R. S. (2014). Natural antiobesity agents bulletin of faculty of pharmacy. *Cairo University*.

[43] Saad B., Azaizeh H., Said O. (2005). Tradition and perspectives of arab herbal medicine: a review. *Evidence-based Complementary and Alternative Medicine*.

[44] Saad B., Zaid H., Shanak S., Kadan S. (2017). *Anti-diabetes and Antiobesity Medicinal Plants and Phytochemicals Safety, Efficacy, and Action Mechanisms*.

[45] Farrington R., Musgrave I. F., Byard R. W. (2019). Evidence for the efficacy and safety of herbal weight loss preparations. *Journal of integrative medicine*.

[46] Näslund E., Hellström P. M. (2007). Appetite signaling: from gut peptides and enteric nerves to brain. *Physiology and Behavior*.

[47] Murphy K. G., Bloom S. R. (2006). Gut hormones and the regulation of energy homeostasis. *Nature*.

[48] Lairon D., Lafont H., Vigne J. L., Nalbone G., Léonardi J., Hauton J. C. (1985). Effects of dietary fibers and cholestyramine on the activity of pancreatic lipase in vitro. *The American Journal of Clinical Nutrition*.

[49] Jamous R. M., Abu-Zaitoun S. Y., Akkawi R. J., Ali-Shtayeh M. S. (2018). Antiobesity and antioxidant potentials of selected Palestinian medicinal plants. *Evidence-based Complementary and Alternative Medicine*.

[50] Herranz-Lopez M., Fernandez-Arroyo S., Perez-Sanchez A. (2012). Synergism of plant-derived polyphenols in adipogenesis: perspectives and implications. *Phytomedicine*.

[51] Kumar P., Bhandari U. (2015). Common medicinal plants with antiobesity potential: a special emphasis on fenugreek. *Ancient Science of Life*.

[52] Saad B., Said O. (2011). Herbal medicine. *Greco-Arab and Islamic Herbal Medicine: Traditional System, Ethics, Safety, Efficacy and Regulatory Issues*.

[53] Salehi B., Ata A., Anil Kumar V. (2019). Antidiabetic potential of medicinal plants and their active components. *Biomolecules*.

[54] Chang H. Y., Wallis M., Tiralongo E. (2007). Use of complementary and alternative medicine among people living with diabetes: literature review. *Journal of Advanced Nursing*.

The article "Anti-Diabesity Middle Eastern Medicinal Plants and Their Action Mechanisms" was published in 2022. Journal: Evid Based Complement Alternat Med.

[55] Kadan S., Saad B., Sasson Y., Zaid H (2013). *In Vitro*Evaluations of cytotoxicity of eight antidiabetic medicinal plants and their effect on GLUT4 translocation. *Evidence-based Complementary and Alternative Medicine*.

[56] Kadan S., Saad B., Sasson Y., Zaid H. (2016). In vitro evaluation of anti-diabetic activity and cytotoxicity of chemically analysed Ocimum basilicum extracts. *Food Chemistry*.

[57] Bnouham M M., Ziyyat A A., Mekhfi H H., Tahri A A., Legssyer A A. (2006). Medicinal plants with potential antidiabetic activity—a review of ten years of herbal medicine research (1990-2000). *International Journal of Diabetes and Metabolism*.

[58] Syed Q. A., Rashid Z., Ahmad M. H. (2020). Nutritional and therapeutic properties of fenugreek (Trigonella foenum-graecum): a review. *International Journal of Food Properties*.

[59] Asadi A., shidfar F., Safari M. (2018). Safety and efficacy of *Melissa officinalis* (lemon balm) on ApoA-I, Apo B, lipid ratio and ICAM-1 in type 2 diabetes patients: a randomized, double-blinded clinical trial. *Complementary Therapies in Medicine*.

[60] Kadan S., Sasson Y., Abu-Reziq R. (2018). *Teucrium polium* extracts stimulate GLUT4 translocation to the plasma membrane in L6 muscle cells. *Advancement in Medicinal Plant Research*.

[61] Saad B., Said O. (2011). The current state of knowledge of arab herbal medicine. *Greco-Arab and Islamic Herbal Medicine: Traditional System, Ethics, Safety, Efficacy and Regulatory Issues*.

[62] Panda A., Jena S., Sahu P. K., Nayak S., Padhi P. (2013). Effect of polyherbal mixtures on the treatment of diabetes. *ISRN Endocrinology*.

[63] Madić V., Petrović A., Jušković M. (2021). Polyherbal mixture ameliorates hyperglycemia, hyperlipidemia and histopathological changes of pancreas, kidney and liver in a rat model of type 1 diabetes. *Journal of Ethnopharmacology*.

[64] Said O., Fulder S., Khalil K., Azaizeh H., Kassis E., Saad B. (2008). Maintaining a physiological blood glucose level with “glucolevel,” a combination of four anti-diabetes plants used in the traditional arab herbal medicine. *Evidence-based Complementary and Alternative Medicine*.

[65] Vaněčková I., Maletínská L., Behuliak M., Nagelová V., Zicha J., Kuneš J. (2014). Obesity-related hypertension: possible pathophysiological mechanisms. *Journal of Endocrinology*.

[66] Hall J. E., da Silva A. A., do Carmo J. M. (2010). Obesity-induced hypertension: role of sympathetic nervous system, leptin, and melanocortins. *Journal of Biological Chemistry*.

[67] Di Chiara T., Argano C., Corrao S., Scaglione R., Licata G. (2012). Hypoadiponectinemia: a link between visceral obesity and metabolic syndrome. *Journal of Nutrition and Metabolism*.

The article "Anti-Diabesity Middle Eastern Medicinal Plants and Their Action Mechanisms" was published in 2022. Journal: Evid Based Complement Alternat Med.

[68] Susalit E., Agus N., Effendi I. (2011). Olive (Olea europaea) leaf extract effective in patients with stage-1 hypertension: comparison with Captopril. *Phytomedicine*.

[69] Mulrow C. D., Chiquette E., Angel L. (2008). WITHDRAWN: dieting to reduce body weight for controlling hypertension in adults. *Cochrane Database of Systematic Reviews*.

[70] Salem M. L., Hossain M. S. (2000). Protective effect of black seed oil from Nigella sativa against murine cytomegalovirus infection. *International Journal of Immunopharmacology*.

[71] Dalli M., Bekkouch O., Azizi S. E., Azghar A., Gseyra N., Kim B. (2021). Nigella sativa L. Phytochemistry and pharmacological activities: a review (2019–2021). *Biomolecules*.

[72] Khan J., Ali A., Balyan P., Bhat E. A. (2022). Role of Nigella sativa as immunomodulator. *InBlack Seeds (Nigella Sativa)*.

[73] Leong X. F., Rais Mustafa M., Jaarin K. (2013). Nigella sativa and its protective role in oxidative stress and hypertension. *Evidence-Based Complementary and Alternative Medicine*.

[74] El-Tahir K. E. H., Al-Ajmi M. F., Al-Bekairi A. M. (2003). Some cardiovascular effects of the dethymoquinonated Nigella sativavolatile oil and its major components *α*-pinene and p-cymene in rats. *Saudi Pharmaceutical Journal*.

[75] Gamboa-Gómez C. I., Rocha-Guzmán N. E., Gallegos-Infante J. A., Moreno-Jiménez M. R., Vázquez-Cabral B. D., González-Laredo R. F. (2015). Plants with potential use on obesity and its complications. *EXCLI Journal*.

[76] Yousfi F., Abrigach F., Petrovic J. D., Sokovic M., Ramdani M. (2021). Phytochemical screening and evaluation of the antioxidant and antibacterial potential of Zingiber officinale extracts. *South African Journal of Botany*.

[77] Sahebkar A., Pirro M., Banach M., Mikhailidis D. P., Atkin S. L., Cicero A. F. G. (2018). Lipid-lowering activity of artichoke extracts: a systematic review and meta-analysis. *Critical Reviews in Food Science and Nutrition*.

[78] Asgary S., Salehizadeh L., Keshvari M. (2018). Potential cardioprotective effects of sumac capsule in patients with hyperlipidemia: a triple-blind randomized, placebo-controlled crossover trial. *Journal of the American College of Nutrition*.

[79] Saad B., Zaid H., Shanak S., Kadan S. (2017). Hypoglycemic and antiobesity polyherbal mixtures. *Anti-diabetes and Antiobesity Medicinal Plants and Phytochemicals Safety, Efficacy, and Action Mechanisms*.

[80] Widmer R. J., Flammer A. J., Lerman L. O., Lerman A. (2015). The Mediterranean diet, its components, and cardiovascular disease. *The American Journal of Medicine*.

The article "Anti-Diabesity Middle Eastern Medicinal Plants and Their Action Mechanisms" was published in 2022. Journal: Evid Based Complement Alternat Med.

[81] Khayyal M. T., el-Ghazaly M. A., Abdallah D. M., Nassar N. N., Okpanyi S. N., Kreuter M. H. (2011). Blood pressure lowering effect of an olive leaf extract (Olea europaed) in L-NAME induced hypertension in rats. *Arzneimittelforschung*.

[82] Guasch-Ferré M., Liu G., Li Y. (2020). Olive oil consumption and cardiovascular risk in U.S. adults. *Journal of the American College of Cardiology*.

[83] Katsiki N., Pérez-Martínez P., Lopez-Miranda J. (2021). Olive oil intake and cardiovascular disease prevention: “seek and you shall find”. *Current Cardiology Reports*.

[84] Perrinjaquet-Moccetti T., Busjahn A., Schmidlin C., Schmidt A., Bradl B., Aydogan C. (2008). Food supplementation with an olive (Olea europaea L.) leaf extract reduces blood pressure in borderline hypertensive monozygotic twins. *Phytotherapy Research*.

[85] de Bock M., Derraik J. G. B., Brennan C. M. (2013). Olive (Olea europaea L.) leaf polyphenols improve insulin sensitivity in middle-aged overweight men: a randomized, placebo-controlled, crossover trial. *PLoS One*.

[86] Said O., Saad B., Fulder S., Amin R., Kassis E., Khalil1 K. (2009). Hypolipidemic activity of extracts from Eriobotrya japonica and Olea europaea, traditionally used in the Greco-Arab medicine in maintaining healthy fat levels in the blood. *The Open Complementary Medicine Journal*.

[87] Shen Y., Song S. J., Keum N., Park T. (2014). Olive leaf extract attenuates obesity in high-fat diet-fed mice by modulating the expression of molecules involved in adipogenesis and thermogenesis. *Evidence-based Complementary and Alternative Medicine*.

[88] Aune D., Giovannucci E., Boffetta P. (2017). Fruit and vegetable intake and the risk of cardiovascular disease, total cancer and all-cause mortality-a systematic review and dose-response meta-analysis of prospective studies. *International Journal of Epidemiology*.

[89] Mink P. J., Scrafford C. G., Barraj L. M. (2007). Flavonoid intake and cardiovascular disease mortality: a prospective study in postmenopausal women. *The American Journal of Clinical Nutrition*.

[90] Chong M. F. F., Macdonald R., Lovegrove J. A. (2010). Fruit polyphenols and CVD risk: a review of human intervention studies. *British Journal of Nutrition*.

[91] Kelley D. S., Adkins Y., Laugero K. D. (2018). A review of the health benefits of cherries. *Nutrients*.

[92] Zheng J., Zhou Y., Li S. (2017). Effects and mechanisms of fruit and vegetable juices on cardiovascular diseases. *International Journal of Molecular Sciences*.

[93] Crowe F. L., Roddam A. W., Key T. J. (2011). Fruit and vegetable intake and mortality from ischaemic heart disease: results from the European Prospective Investigation into Cancer and Nutrition (EPIC)-Heart study. *European Heart Journal*.

The article "Anti-Diabesity Middle Eastern Medicinal Plants and Their Action Mechanisms" was published in 2022. Journal: Evid Based Complement Alternat Med.

[94] Good C. K., Holschuh N., Albertson A. M., Eldridge A. L. (2008). Whole grain consumption and body mass index in adult women: an analysis of NHANES 1999-2000 and the USDA pyramid servings database. *Journal of the American College of Nutrition*.

[95] Ali M. Y., Sina A. A. I., Khandker S. S. (2020). Nutritional composition and bioactive compounds in tomatoes and their impact on human health and disease: a review. *Foods*.

[96] Linnewiel H. K., Shefer I., Raz G. (2016). *Tomato based supplement supports cardiovascular health The FASEB Journal*.

[97] Burton-Freeman B. M., Sesso H. D. (2014). Whole food versus supplement: comparing the clinical evidence of tomato intake and lycopene supplementation on cardiovascular risk factors. *Advances in Nutrition*.

[98] Sesso H. D., Wang L., Ridker P. M., Buring J. E. (2012). Tomato-based food products are related to clinically modest improvements in selected coronary biomarkers in women. *Journal of Nutrition*.

[99] Cheng H. M., Koutsidis G., Lodge J. K., Ashor A., Siervo M., Lara J. (2017). Tomato and lycopene supplementation and cardiovascular risk factors: a systematic review and meta-analysis. *Atherosclerosis*.

[100] Chen J. P., Chen G. C., Wang X. P., Qin L., Bai Y. (2017). Dietary fiber and metabolic syndrome: a meta-analysis and review of related mechanisms. *Nutrients*.

[101] Gervasi T., Barreca D., Laganà G., Mandalari G. (2021). Health benefits related to tree nut consumption and their bioactive compounds. *International Journal of Molecular Sciences*.

[102] Jamshed H., Sultan F. A. T., Iqbal R., Gilani A. H. (2015). Dietary almonds increase serum HDL cholesterol in coronary artery disease patients in a randomized controlled trial. *Journal of Nutrition*.

[103] Kingwell B. A., Chapman M. J., Kontush A., Miller N. E. (2014). HDL-targeted therapies: progress, failures and future. *Nature Reviews Drug Discovery*.

[104] Yu Z., Malik V. S., Keum N. (2016). Associations between nut consumption and inflammatory biomarkers. *The American Journal of Clinical Nutrition*.

[105] Scalbert A., Manach C., Morand C., Remesy C., Jimenez L. (2005). Dietary polyphenols and the prevention of diseases. *Critical Reviews in Food Science and Nutrition*.

[106] Pereira D. M., Valentão P., Pereira J. A., Andrade P. B. (2009). Phenolics: from chemistry to biology. *Molecules*.

[107] Pandey K. B., Rizvi S. I. (2009). Plant polyphenols as dietary antioxidants in human health and disease. *Oxidative Medicine and Cellular Longevity*.

[108] Gao S., Hu M. (2010). Bioavailability challenges associated with development of anti-cancer phenolics. *Mini-Reviews in Medicinal Chemistry*.

The article "Anti-Diabesity Middle Eastern Medicinal Plants and Their Action Mechanisms" was published in 2022. Journal: Evid Based Complement Alternat Med.

[109] Rabkin R. (2003). Diabetic nephropathy. *Clinical Cornerstone*.

[110] Brownlee M. (2001). Biochemistry and molecular cell biology of diabetic complications. *Nature*.

[111] Sheetz M. J., King G. L. (2002). Molecular understanding of hyperglycemia’s adverse effects for diabetic complications. *JAMA*.

[112] Cooper M. E., Gilbert R. E., Epstein M. (1998). Pathophysiology of diabetic nephropathy. *Metabolism*.

[113] Brands M. W., Fitzgerald S. M., Hewitt W. H., Hailman A. E. (2000). Decreased cardiac output at the onset of diabetes: renal mechanisms and peripheral vasoconstriction. *American Journal of Physiology—Endocrinology And Metabolism*.

[114] Zhou L. T., Zhang Z. J., Cao J. Y. (2021 Jun). The unique molecular mechanism of diabetic nephropathy: a bioinformatics analysis of over 250 microarray datasets. *Clinical kidney journal*.

[115] Mapanga R. F., Musabayane C. T. (2010). The renal effects of blood glucose-lowering plant-derived extracts in diabetes mellitus—an overview. *Renal Failure*.

[116] Dwivedi C., Daspaul S. (2013). Antidiabetic herbal drugs and polyherbal formulation used for diabetes: a review. *The Journal of Phytopharmacology*.

[117] (2003). WHO Diet, nutrition and the prevention of chronic diseases. *Report of a Joint FAO, WHO Expert Consultation. WHO Technical Report Series*.

[118] Wang Y., Gallegos J. L., Haskell-Ramsay C., Lodge J. K. (2021). Effects of chronic consumption of specific fruit (berries, citrus and cherries) on CVD risk factors: a systematic review and meta-analysis of randomised controlled trials. *European Journal of Nutrition*.

[119] Zaid H., Saad B. (2013). State of the art of diabetes treatment in greco-arab and islamic medicine. *Bioactive Food as Dietary Interventions for Diabetes*.

